# The Feature Recognition of Motor Noise Based on the Improved EEMD Model

This article has been retracted.

**DOI:** 10.1155/2022/9172719

**Published:** 2022-08-18

**Authors:** Qing Liao, Long Li, Jiaqi Luo

**Affiliations:** ^1^Intelligent Manufacturing College of Wuhan Guanggu Vocational College, Wuhan 430079, Hubei, China; ^2^Wuhan Technology and Business University, Wuhan 430065, Hubei, China

## Abstract

The noise generated by the machine is closely related to the running state of the machine, so the product can be effectively detected by analyzing the noise signal. The noise identification and control methods based on the EEMD model are widely used in motor noise control. However, the EEMD only considers the influence of noise amplitude on the decomposition results, and the added white noise cannot be completely neutralized. In this paper, an improved EEMD method is proposed by analyzing the influence of the maximum frequency on the decomposition results, in which the noise with different maximum frequency and amplitude is added to decompose the signal, and the decomposition effect is judged by the orthogonality coefficient of the decomposition result. Finally, the simulation signal and the measured signal are compared and analyzed, and the results show that the improved EEMD method has some advantages over the original method in suppressing mode confusion and fault diagnosis.

## 1. Introduction

The machine will not only produce vibration but also produce noise; the noise generated by the machine during operation is closely related to the running state of the machine [1, 2]. Most manufacturers have certain requirements for the noise level of the machine, so the online detection of motor noise is a research hotspot. By analyzing and identifying the noise signal, it can not only eliminate the unqualified motor in the production line but also analyze the fault of the product. The traditional methods mainly include three kinds, namely, the subjective identification method, the near-field test method, and the step-by-step operation method. These methods cannot quantitatively describe the noise, and excessive dependence on practical experience also makes the recognition accuracy of the algorithm low [3, 4]. In recent years, the noise identification and control method based on the EEMD model has been widely used in motor noise control. However, the EEMD method has two disadvantages: the EEMD method only considers the influence of noise amplitude on the decomposition results, and the added white noise cannot be completely neutralized, so the improvement of the EEMD model is of great significance to grasp the running state of mechanical equipment effectively.

Aiming at the problem of motor noise, scholars have carried out a lot of research. The noise mechanism and control method of the motor are studied in reference [5, 6], the criteria for evaluating the noise performance of the motor are proposed, as well as the method of identifying the noise source of the motor and the measure of reducing the electromagnetic noise, are proposed. It is pointed out in the reference that the main component of motor noise is electromagnetic noise [7], and the structure noise accounts for a large proportion at high speed, while the ventilation noise produced by the fan can be ignored. At the same time, a method of reducing electromagnetic noise and structural noise is proposed. The mechanism of motor noise is analyzed in reference [8], and it is suggested that the rigidity of parts should be considered in the design of the motor to avoid resonance. Taking a switched reluctance motor as the research object, the natural mode and frequency of the motor are calculated by using the finite element method, and an approximate formula for predicting the natural vibration modal frequency is proposed [9]. A fast and accurate noise prediction method is proposed in reference [10], in which the acceleration of the stator can be calculated by rotor position and voltage waveform, and the noise caused by the stator can be calculated by the boundary element method. A hybrid prediction method for motor noise is proposed in reference [11], and the performance of motor noise is evaluated under various operating conditions. The results show that this method can provide a reliable prediction for the main noise during acceleration. To sum up, for the study of noise source identification of mechanical equipment with large noise problems, scholars have obtained certain research results, and the sound source identification can be accurately studied through signal processing. However, the research on the identification of motor noise sources has achieved relatively few results, which needs further research.

Firstly, the problem of motor noise feature recognition is described, the relevant model that is in combination with the actual situation is established, and the relevant assumptions are given. Then, an improved EEMD method is proposed, which analyzes the influence of noise maximum frequency on decomposition results. Finally, the practicability of the proposed method is verified by experiments.

## 2. Problem Description and Hypothesis

The movement of machine parts will inevitably produce vibration, which will then radiate noise. The noise generated by the machine during operation is closely related to the running state of the machine; when the movement of machine parts and the mutual movement of parts change, the noise signal of the machine will also change. The abnormal noise is associated with a specific fault; the running state of the machine can be monitored and fault-diagnosed through the analysis of the noise signal. Before analyzing the problem, we should describe the problem first, and then the model of problems should be solved.

### 2.1. Noise Generation

The motor noise is a complex problem, which can be divided into three categories according to the source of noise: the electromagnetic noise, the aerodynamic noise, and the mechanical noise [12]. The aerodynamic noise of the motor system with natural air cooling or forced liquid cooling can be ignored. In the motor noise, the electromagnetic noise accounts for the main contribution, and the contribution of mechanical noise is the second.

#### 2.1.1. Electromagnetic Noise

The electromagnetic noise is mainly caused by phase imbalance and magnetic saturation; when the rotor of the motor is unbalanced, a force biased towards the rotation center will be generated due to the effect of centrifugal force. The unbalanced force is mainly related to the rotation speed, eccentric mass, and eccentricity, which will affect the reliability of the motor rotor and make the motor work abnormally. The noise produced by rolling bearings is one of the main noises in the mechanical noise of the motor, and the bearing noise is generally considered to be an integral multiple of the product of bearing rotation frequency and the number of rollers [13]. When there are problems such as insufficient lubricating oil and poor oil in bearing lubrication, the noise is more obvious because of the impact and mechanical friction.

#### 2.1.2. Mechanical Noise

The mechanical noise in the motor is mainly caused by the imbalance of the bearing and rotor, which is related to the selected material and mass load assembly process. The mechanical noise generated during the operation of the machine is mainly divided into four categories, which are the movement of the machine parts themselves, such as the contact between the machine parts, the transmission of force between the machine parts, and the interaction between the machine parts and the periphery.

Firstly, the movement of the machine parts themselves produces noises. The parts such as shafts, gears, and clutches produce noises due to the excitation of unbalanced centrifugal force, while the reciprocating parts such as pistons and punches produce noises due to the excitation of inertial force. Secondly, the contact between the parts of the machine produces sound. In rolling bearings, friction wheel mechanisms, and belt wheel mechanisms, the interaction between the two error surfaces makes sound. Then, the transmission of forces between the machine parts produces sound. The mechanical transmission mechanism produces noise due to the uneven transmission of force, impact, friction, and assembly error, and the hydraulic transmission mechanism produces noise due to flow fluctuation [14]. Finally, the interaction between the machine parts and the periphery will produce sound. The parts such as the cylinders, pipelines, and propellers make noises due to the separation of turbulence.

### 2.2. Description of the Problem

In the analysis of motor noise, we need to describe and mathematise the problem first. Based on the basic theory of acoustics, a simplified model is proposed in this paper, in which each machine is regarded as a point source, and the radiated sound field is calculated according to the sound field radiated by the point source in the free sound field. It is assumed that there are many mechanical noise sources in the actual production plant, and there are many other uncertain sounds at the same time, such as the voice of people and the accidental collision between objects [15]. The actual number of sound sources is a lot, but considering that many of them are secondary or negligible, they can be treated as noise.

It is assumed that the microphone is used to measure the noise source in the factory. Firstly, a proper coordinate system is established to record the position of the noise source and the microphone, and the sound emitted by the sound source is calculated according to the radiated sound field of the point sound source. The signals received by the microphone include sound signals and background noises from various sound sources, and the estimation of the transfer matrix between the sound source and the microphone can be obtained by obtaining the position and number of the sound source.

### 2.3. Basic Assumptions

The noise generated by the machine during operation is closely related to the running state of the machine, and the state monitoring of the machine can be carried out by noise signal analysis. In practical production, the useful information in sound is often submerged in a very complex background noise, which seriously affects the accuracy and reliability of fault diagnosis. How to obtain the fault noise source position of the equipment to be diagnosed and extract the fault signal from the mixed signal is the key to improving the practicability of acoustic fault diagnosis technology. Due to the complexity of the actual field environment, some simplifications are needed, and the assumptions made in this paper are as follows.

Firstly, the sound signal from the source is a stationary random signal, and the noise in the measurement process is the additive Gaussian white noise. Secondly, the signal sources are considered additive at a certain time. Thirdly, the signals are independent of each other. Fourthly, the mechanical noise sources are regarded as point sources, and the radiated sound field is a free sound field. Finally, each signal source is independent of the other, and the signals are added instantaneously.

## 3. Motor Noise Source Identification Method and Improvement

A motor is a kind of rotating machinery with a relatively complex structure, whose noise signal is a typical nonstationary time-varying signal with a wide frequency band and complex frequency components. In view of the complexity of motor noise signal and the limitation of current noise source identification methods, the EEMD model is improved, and an improved signal processing method is proposed to analyze the motor noise signal. The IMF decomposed by the EEMD is used as the input of the FastICA algorithm, which can effectively suppress the deficiency of modal aliasing in the EMD method.

### 3.1. The EEMD Method

As the core of the EEMD method, the EMD can decompose the nonstationary signal into two parts: one part is a series of intrinsic mode functions with zero mean, and the other part is an eigenvalue term. Each IMF component must satisfy two basic conditions [12]: one is that the number of extreme points and zeros of the signal must be equal, and the other is that the average value of the upper and lower envelope of the signal should be zero.

Among the defects of the EMD method, the modal mixing is the most important. In order to reduce this phenomenon, the EEMD method is proposed, in which the white noise is added to the measured signal. The distribution characteristics of the original signal extreme points are changed to make the distribution more uniform, which can effectively suppress the mode aliasing. At the same time, this method applies the multidecomposition results to the lumped average calculation, which can reduce the chance of mode aliasing. The steps of the method are shown in Figure 1.

Firstly, the white noise should be added to the original signal and the newly generated signal should be decomposed by the EMD. Then, different white noises with fixed amplitude are added, and the above steps are repeated. Finally, the decomposition results can be obtained by lumping and averaging the components of the same order.

### 3.2. FastICA Method

Assuming that the three machines make simultaneous sounds in one room, the signal *x*_*i*_(*t*)(*i*=1,2,3) recorded with three microphones at different locations is the linear weighted sum of three speech signals, as shown in formulas (1)–(3).

(1) $$\begin{array}{c} x_{1}\left(t\right)=h_{11}s_{1}\left(t\right)+h_{12}s_{2}\left(t\right)+h_{13}s_{3}\left(t\right), \end{array}$$

(2) $$\begin{array}{c} x_{2}\left(t\right)=h_{21}s_{1}\left(t\right)+h_{22}s_{2}\left(t\right)+h_{23}s_{3}\left(t\right), \end{array}$$

(3) $$\begin{array}{c} x_{3}\left(t\right)=h_{31}s_{1}\left(t\right)+h_{32}s_{2}\left(t\right)+h_{33}s_{3}\left(t\right), \end{array}$$

where *h*_*ij*_ represents the weight coefficient, which is related to the microphone position and the distance between the microphone and the speaker.

This problem of estimating the original speech signal by recording the signal is the cocktail party problem, whose signal mixing is shown in Figure 2.

If the three source signals are independent of each other, the blind signal processing algorithm can be used to recover the source signal from the mixed signal. The recovered signal is very similar to the original signal, but the order of the recovered signal is usually inconsistent with the original signal. This problem generally does not affect the separation and identification of noise sources because it is easy to determine the specific signal source according to the noise mechanism of the source signal and the corresponding prior knowledge.

In this paper, the mathematical language is used to describe the ICA problem. Suppose *x* is an m-dimensional observation signal vector, which is composed of multiple independent source signals. Therefore, the model can be expressed by formula (4), and its matrix form is shown in formula (5).

(4) $$\begin{array}{c} x=Hs, \end{array}$$

(5) $$\begin{array}{c} \left[\begin{array}{c} x_{1}\left(t\right)\\ \ldots \\ x_{m}\left(t\right) \end{array}\right]=\left[\begin{array}{c} \begin{array}{ccc} h_{11} & \ldots & h_{11} \end{array}\\ \begin{array}{cc} \ldots & \ldots \end{array}\\ \begin{array}{ccc} h_{11} & \ldots & h_{11} \end{array} \end{array}\right]\left[\begin{array}{c} s_{1}\left(t\right)\\ \ldots \\ s_{m}\left(t\right) \end{array}\right], \end{array}$$

where *x* represents the observation signal vector, H represents the signal matrix, and *s* represents the unknown zero-mean independent source signal.

It can be seen from formula (6) that the observed data at a certain time can be obtained. The problem to be solved in blind source separation is that when the source signal and the mixed signal are unknown, a certain priori-knowledge should be added to estimate a matrix, so the formula (6) can be obtained through the linear transformation of *x*.

(6) $$\begin{array}{c} y=Px, \end{array}$$

where *y*=(*y*_1_, *y*_2_,…,*y*_*n*_)^*T*^ represents the estimate of the source signal, and P represents the separation matrix.

Compared with the traditional algorithm, the FastICA method has faster convergence speed, which does not need to choose step size parameters, indicating that the algorithm is easier to use. In this paper, the FastICA method based on maximum negative entropy is adopted, which takes maximum negative entropy as a search direction. The independent sources can be extracted sequentially, which fully reflects the linear transformation idea of projection pursuit. The iteration of the algorithm is shown in formulas (7) and (8).

(7) $$\begin{array}{c} W^{*}=\frac{W-\left[E\left\{Xg\left(W^{T}X\right)\right\}-\beta W\right]}{\left[Eg^{\prime }\left(W^{T}X\right)-\beta \right]}, \end{array}$$

(8) $$\begin{array}{c} W=\frac{W^{*}}{\left\|W^{*}\right\|}, \end{array}$$

where *W*^*∗*^ is a new value of *W*; the regularization of parameters can improve the robustness of the solution.

### 3.3. The Improved EEMD Method

It can be seen that the Newton iteration method is adopted to solve the problem, and its iteration formula is shown in the following formula:

(9) $$\begin{array}{c} x_{k+1}=x_{k}-\frac{f\left(x_{k}\right)}{f^{\prime }\left(x_{k+!}\right)}. \end{array}$$

In the FastICA algorithm, formula (10) is obtained according to formula (9), and then the value of W is estimated. When f(a) = 0 and *f* '(a) is not equal to 0, formula 9is the second-order convergent. In order to further improve the convergence speed of Newton iteration, the following improved iteration formula is given:

(10) $$\begin{array}{c} z_{n+1}=x_{k}-\frac{f\left(x_{n}\right)}{f^{\prime }\left(x_{n+1}\right)}, \end{array}$$

(11) $$\begin{array}{c} x_{n+1}=x_{n}-\frac{2f\left(x_{n}\right)}{\left(f^{\prime }\left(x_{n}\right)+f^{\prime }\left(z_{n}+1\right)\right)}, \end{array}$$

where *f*(*x*_*n*_) represents the objective function and *x*_*n*+1_ represents the solution to the problem.

Aiming at the shortcomings of the measurement signal in the noise source separation and identification, a method that is based on the improved EEMD is proposed. The motor noise signal of a single channel is analyzed and studied, and the basic process is shown in Figure 3.

The motor noise signal has two characteristics: one is nonstationary, and the other is the uncertainty of the noise source. Aiming at the problems of motor noise, the EEMD method can decompose the motor noise signal into a series of IMF, and then the IMF decomposed by EEMD is used as the input of the FastICA algorithm. The improved EEMD method makes the advantages of the two methods complement each other, which can suppress the deficiency of modal aliasing in the EMD method so that the improved EEMD method has better performance.

## 4. System Performance Analysis

Since the proposed method will eventually be applied to motor noise signal processing, the performance of the improved EEMD method must be analyzed before application. The EEMD method is used to analyze and process the measured noise signal, and the processing results are compared with those of the proposed method in this paper.

### 4.1. Influence of SNR

In order to research the influence of the SNR on the recognition effect, the white noise with the different SNR is added to the mixed noise. The noise source separation simulation is repeated 100 times for each SNR, and the average value of the simulation is taken as the result. The absolute value of the correlation coefficient with the source signal is counted, and the results are shown in Figure 4.

It can be seen from Figure 4 that the correlation coefficient of the noise source increases with the increase of the SNR. In general, the correlation coefficient of the improved EEMD is always greater than that of the EEMD, indicating that the recognition effect of the improved EEMD is always significantly higher than that of the EEMD. The difference in correlation coefficients between the two methods decreases with the increase of the SNR, which indicates that the recognition effect of the improved EEMD is significantly higher than that of the EEMD when the SNR is low, and the recognition effect of the improved EEMD and the EEMD is similar when the SNR is high. The correlation coefficient of the two algorithms above 20 dB is greater than 0.6, which indicates that they have good anti-interference ability.

### 4.2. Effect of Sampling Frequency

In order to research the effect of sampling frequency on noise source recognition, the white noise is added to the mixed signal while the frequency range of the noise is 10000 Hz∼20000 Hz. Each simulation is repeated 100 times; the average value of each simulation is taken as the result, and the performance comparison at different sampling frequencies is shown in Figure 5.

It can be seen from Figure 5 that the correlation coefficient of the improved EEMD is greater than that of the EEMD under the same noise source signal, which indicates that the recognition effect of the improved EEMD is better than that of the EEMD. With the increase of sampling frequency, the correlation coefficient difference between the EEMD and the improved EEMD decreases, which indicates that the recognition effects of the two recognition methods are the same under high sampling frequency.

### 4.3. Quantitative Analysis of Fault Frequency

Both the methods suppress modal confusion to some extent. In order to better illustrate the advantages of the improved EEMD method, the envelope spectra of the four components of the decomposition results are calculated, and the fault frequency in the envelope spectrum is quantitatively analyzed by formula 12.

(12) $$\begin{array}{c} \gamma =\frac{A_{f}}{\sum A_{a}}, \end{array}$$

where *A*_*f*_ represents the failure frequency and *A*_*a*_ represents the analysis frequency.

The results are shown in Figure 6; the results show that the fault frequency spectrum line of the original EEMD method is lower than the amplitude of the interference frequency in the fourth component, which will cause interference to the fault judgment. The fault frequency amplitude of the improved EEMD method is still greater than the interference frequency, which can accurately determine the fault; it is clear that the improved EEMD method has a good effect.

## 5. Conclusion

Firstly, the problem of motor noise feature recognition is described, and a simplified model based on the basic theory of acoustics is proposed, in which the relevant assumptions are given in combination with the actual situation. Then, the influence of the maximum frequency on the decomposition results is analyzed in this paper, in which the problem of the EEMD method can be solved. Aiming at the complexity of the motor noise signal, an improved signal processing method is proposed to analyze the motor noise signal, which can realize the separation and identification of the sound source. Finally, the EEMD method is used to analyze and process the measured noise signal, and the processing results are compared with those of the improved EEMD. The results show that the separated signal obtained by the improved EEMD method can remove a lot of noise, and the recognition effect of the improved EEMD method is better than that of the EEMD. The fault frequency amplitude of the improved EEMD method is greater than the interference frequency, which is more conducive to accurate fault judgment. Therefore, the improved EEMD method has some advantages over the original method in suppressing mode confusion and fault diagnosis.

## Figures and Tables

**Figure 1:** The flow chart of EEMD.

**Figure 2:** The FastICA model.

**Figure 3:** Basic flow of the improved EEMD.

**Figure 4:** The influence of SNR.

**Figure 5:** The effect of sampling frequency.

**Figure 6:** The fault frequency value.

## Data Availability

The dataset can be accessed upon request.
